# Reducing Requirements Ambiguity via Gamification: Comparison with Traditional Techniques

**DOI:** 10.1155/2022/3183411

**Published:** 2022-07-18

**Authors:** Hafsa Shareef Dar, Salma Imtiaz, Muhammad IkramUllah Lali

**Affiliations:** ^1^Department of Computer Science & Software Engineering, Faculty of Basic & Applied Sciences IIU Islamabad, Islamabad, Pakistan; ^2^Department of Software Engineering, Faculty of Computing & IT, University of Gujrat, Gujrat City, Pakistan; ^3^Department of Information Sciences, University of Education Lahore, Jauharabad Campus, Lahore, Pakistan

## Abstract

Requirements elicitation is one of the most significant activities of requirements engineering (RE) process. Poorly specified requirements can lead to a failed project. Various elicitation techniques are used to elicit requirements from the users and other stakeholders, each having its own pros and cons. Lack of user engagement, less user involvement, textual nature of the requirements, time taking process are some of the major problems that make it difficult to perform elicitation via traditional techniques. Moreover, these problems further create other challenges such as ambiguity, inconsistency, and incompleteness in requirements. Currently, researchers have focused on reducing ambiguity in requirements with the help of different techniques such as natural language processing techniques, requirement templates, and formal methods; however, these techniques work on reducing ambiguity during specification or from specified requirements. One of the “young' and exciting way of engaging users in requirements elicitation of a system is “Gamification', which helps in user engagement into the system. We intend to discover how gamification helps in reducing ambiguity by engaging stakeholders in an interactive manner. In this review study, we have reviewed traditional techniques used to detect and reduce requirements ambiguity. On the contrary, we have also presented the significance of gamification in requirements elicitation and the popular but effective game elements used in similar systems. Furthermore, this study highlights the significance of using gamification in requirements elicitation, which is beneficial to software development team as well as the users involved in the system.

## 1. Introduction

Requirements are gathered during requirements elicitation using different methods [1], but this activity has many challenges such as lack of requirements understanding, less user involvement, and more user expectation from the system under development [2]. These challenges create major problems in the system in later stages. However, the requirements must be specified with great care to avoid any kind of ambiguity during software development.

In requirements engineering (RE), ambiguity is defined as “*having multiple interpretations despite the readers knowledge of the RE context*”[3]. Literature is evident that ambiguity in requirements is a more intractable problem than the other problems in requirements like misunderstood and incomplete requirements [4] because requirements are specified in natural language (NL) [5, 6]. One way to avoid ambiguity is specification of requirements in formal languages. The formal languages are based on mathematical evaluations to strictly define the syntax and semantics of the language and are helpful in equivalence verification of the requirements between specification and implementation phase. Writing formal specifications is a complex and time taking process and requires expertise. Although formal and constrained languages are proposed due to their structure to avoid ambiguity, they lack the depth of NL in expressing the concept [7].

The NL comes with the two extremely significant merits, that is, understandability and acceptance, unlike constrained and formal languages, it is prone to ambiguity that results in incompleteness, inconsistency, and misunderstanding in requirements specifications [8]. These misunderstandings occur due to the constraints of NL expressions inferred by the man-made judgments of the real scenarios. These misunderstandings later pass on to other software development phases [9]. Requirements are expressed and documented in NL in most of the RE artefacts, in which ambiguity is an active challenge, and reducing it is one complex task [10]. Understanding the nature and identifying the source of ambiguity helps in reducing its effect during software development. The researchers have classified different types of ambiguity, among which one notable taxonomy on ambiguity classification is given by Berry [11, 12].

The rest of the paper is organized in different sections.  Section 2 presents a background on gamification and game elements, Section 3 presents methodology of the paper, detailed review of the literature covering ambiguity in elicitation, gamification in elicitation, and gaming elements for requirements elicitation is presented in Section 4. Section 5 presents findings of the review, whereas Section 6 presents conclusion and future work.

### 1.1. Background

#### 1.1.1. Lexical Ambiguity

This type of ambiguity occurs when a word has more than one meaning [13, 14]. It is divided into two parts homonymy and polysemy. Homonymy arises as a word with distinct meanings along with etymologies (same spellings but different meanings) [15], e.g., bank: “world bank means a depository of financial institution” and “sloping land.” Polysemy word consists of several meanings that are interrelated but etymology or having different contexts [14] i.e., word “green” may represent green or a fruit that is unripe [16]. Previously, some research has been done on lexical expressions to lead other types of requirements' ambiguity, but lexical ambiguity lacks research [17].

#### 1.1.2. Syntactic Ambiguity

This is also known as structural ambiguity which arises due to parsing of a sentence in multiple ways, having different meanings [15, 18], for example, a sentence “*I saw a girl with the binoculars*” can be parsed into two different meanings, the girl has binoculars, or I used binocular to see the girl. It is further divided into attachment ambiguity [14]. Attachment ambiguity refers to the doubt of attaching a clause or part of sentence to the other part of the sentence [19].

Nocuous and innocuous ambiguities have been focused in RE [20]. Moreover, previous studies have also discussed the misplaced use of “also”[21] and “only”[22] cues as part of syntactic ambiguity.

#### 1.1.3. Semantic Ambiguity

This type of ambiguity arises when predicate logic has multiple interpretations of the sentence without any lexical or syntactic ambiguity [15]. Under this ambiguity, a sentence can be translated into more than one expression [23]. Coordination, scope, and anaphoric ambiguity are type of semantic ambiguity [14]. Coordination ambiguity arises on the use of more than one conjunction with a modifier in a sentence [19].

Scope ambiguity generally occurs when the words such as “many, some, and each” are used because these words change the scope of a sentence [24]. Anaphoric ambiguity occurs when there is more than one possibility of referring to the word that was mentioned earlier in the sentence [25]. Quantifiers and “all” are the cues of semantic ambiguities [26]. Other cues are “plurals”[27]. It has also been identified in previous studies that semantic ambiguity is not considered in linguistic classification [21], which includes the cues of syntactic ambiguity.

#### 1.1.4. Pragmatic Ambiguity

This type of ambiguity arises due to the uncertainty of human contextual knowledge and common-sense knowledge [13, 18]. Pragmatic ambiguity focuses on requirements context and the meaning [14, 15], including the knowledge of the reader. The readers may have different backgrounds and interpretation of requirements.

#### 1.1.5. Language Errors

Language errors can occur due to poor grammar of sentence [17, 18]. Language errors are considered as a separate class of ambiguity.  Figure 1 show types and subtypes of NL ambiguity.

There are some other classifications of ambiguity including intentional and nonintentional [7], nocuous and innocuous [17], acknowledged and unacknowledged [20]. However, not all ambiguities are considered harmful; the intentional ambiguity is helpful in providing flexibilities in design and implementation phases [10].

In past studies, different natural language processing (NLP) techniques, tools, and methods have been discussed to address ambiguity identification, extraction, removal, and management [3]. Many approaches for ambiguity identification and detection of requirements written in NL are proposed [13]. Requirements written in NL tend to be ambiguous, thus preprocessing of Software Requirements Specifications (SRS) document along with NLP techniques is required to help identify and resolve ambiguity [28]. However, manual ambiguity resolution of software requirements is time consuming, error prone, and costly process [29, 30]. Therefore, the researchers have introduced more interactive solutions to involve stakeholders in the process of RE and requirements elicitation. One of those interactive solutions is “gamification.”

#### 1.1.6. Gamification

Gamification is a method to enhance motivation and involvement of user in the system. In elicitation, gamification has been used in recent years [31–33] with a focus to involve and engage users for the purpose of gathering requirements. There are limited studies present previously that focuses on acquiring unambiguous requirements from the user [34–36]. The term “Gamification” was originated in digital media industry in 2008 and adopted worldwide in 2010 [37]. The term is consistently used by industry players and published in conferences and hence has gained much popularity [5, 38]. It consists of fun gaming elements like video games that are meant for entertaining the users. Gamification is an informal term for enhancing user engagement and experience of gaming elements in nongaming systems [39].

According to the Cambridge Advanced Learner's Dictionary and Thesaurus published by the Cambridge University Press [40], it is defined as “*the practice of making activities more like games in order to make them more interesting or enjoyable*.” Similarly, the Oxford Learner's Dictionary published by the Oxford University Press [41], defined it as “*the use of elements of game-playing in another activity, usually in order to make that activity more interesting*.” The formal definitions indicates that gamification is a process of making gaming activities more interesting, but the effectiveness of gamified systems majorly rely on the way they help the users to achieve their goals [42]. Other similar concepts to gamification are game layers, behavioural games, applied gaming, ludic qualities, storyfication, taskification, gamenics theory, and includification.

#### 1.1.7. Game Elements in Requirements' Elicitation

Gamification is the use of game elements in nongaming contexts [43]. According to the literature [44], the contributors involved in gamification extensively agree that it is a significant approach when used in nongaming contexts. Generally, it is recommended in those systems where boredom, passiveness, and repetition are influential factors. Gamification uses interactive features to motivate and encourage [45] the end-users to participate [46] in the system using game elements and mechanics [43]. It makes boring task enjoyable and interesting [47, 48] by using fun game elements.

Digital games are different as those of gamification [49]. A digital game is more of a formal system based on rules, having measurable outcome depending upon the effort put by the player(s) [50]. The game elements in gamification are used to enhance user engagement in the system.  Table 1 shows the difference between digital games and gamification.

In a digital game, rules and objectives are the driving forces, on the contrary, game elements like rewards and points make the system interesting and enjoyable. The result in game is either winning or losing of players, whereas losing is not an option in the gamification because it tends to encourage the players. Digital games are expensive due to their complex structures, but gamification is not expensive and not a complex medium. Gamification use game elements to solve business problems rather than creating games [51]. In previous studies, these game elements are also described as “ten ingredients of great games.” These game elements are avatars, 3D environments, ranks and levels, reputation, feedback, economies and marketplace, rule-based competition, teams, parallel configurable communication systems, and time pressure [52]. User roles such as designer or user, also play a vital role in perceiving these elements. Hence, the elements are taken as important building blocks of the system.

The literature has discussed other commonly used game elements such as scores and points [53], badges [54], leaderboard [51], awards, rewards, ranks, levels, quests, bets, avatars [54, 55], and stories [49, 56].  Table 2 provides known gaming elements and their description.

Although there are multiple game elements present in the literature, previous studies reveal that the points, badges [57] and voting systems [54] are the most used ones. In some gamified systems, single game element is used to gain some learning experience [44]. These elements are categorized based on their motivational significance and structural characteristics [42], yet this categorization does not help the designer to decide which pattern works well to fulfil user needs, and as a result, they end up choosing Points Badges Leaderboard (PBL) [46] due to their easy implementation in system. A gamified system possesses three types of elements attached to it, including rules, goals, and feedback [49]. First, to play a fair game, easy and clear rules are assigned. Second, attractive and achievable goals are set, the player uses the system with some motive. In last, a good feedback system must be present to provide feedback to the player.

Gamification uses narrative context due to which user can relate to real-life examples more easily than the abstract concepts. Currently, due to fun attributes involved in the system, gamification has grabbed attention in many applications. It is also used in software development to elicit user needs and express user goals [58]. The requirements are an integral part of the system [36] and hence require user's attention as they must elaborate system's behaviour and functionalities [59]. In RE, gamification is applied to requirements elicitation, negotiation, prioritization, validation, and specification. However, requirements specification and validation are the least discovered areas in gamification.

Requirements ambiguity is a huge problem in NL that arise due to unclear system understanding [2]. There is a limited work present which focuses on getting unambiguous and clear requirements [34, 36]. Similarly, a small number of studies have discussed requirements ambiguity in elicitation [1, 34, 60]. Participation in a gamification platform is what results in unambiguous requirements from multiple stakeholders. The aim behind conducting this study is to review existing techniques of ambiguity reduction and gamification in requirements elicitation. The outcome of this review would be helpful to propose a gamification tool for acquiring unambiguous requirements from the users by making them part of a process and system. This research work is a part of PhD thesis on reducing ambiguity in requirements elicitation via gamification. The initial idea and software design of the proposed tool has been published in RE'20 [60, 61].

## 2. Methodology

The purpose of this review is to present an overview on traditional requirements ambiguity identification, detection, and reduction techniques, usefulness of gamification technique to reduce ambiguity during requirements elicitation and identification of well-suited game elements for requirements elicitation. However, the methodology of this study is review based. Firstly, the traditional techniques on NL requirements' ambiguity, and gamification in requirements elicitation were studied and reviewed. Second, the popular and useful game elements discussed in literature were reviewed and shortlisted in terms of frequency of their usage in each selected study.  Figure 2 shows the methodology of this review in detail.

### 2.1. Review of Existing Techniques

#### 2.1.1. Related Work on Ambiguity in Requirements' Elicitation

According to literature [17], ambiguity occurs because of the difference between customers' articulation of unit of information and the meaning assigned to it by the analyst. The articulation of unit of information means any fragment or set of words of a sentence in spoken form, usually articulated by the user. There are two types of information: one is about system needs and the other is about domain aspects of the system. Although, NL is used for requirements specification [62], yet requirements in English may have issues of ambiguity. Ambiguity in NL requirements is handled using three approaches, namely ambiguity detection, ambiguity reduction, and ambiguity removal after detection [3, 63, 64].

Similarly, to document requirements in NL, a system was developed to check validity and lexical ambiguity of written requirements [5]. The system works to check requirements validity and ambiguity in requirements. For this purpose, the algorithm was designed and implemented. The authors concluded that any kind of ambiguity might be present in the sentence other than the lexical ambiguity. A tool for detecting lexical and syntactic ambiguity in words and sentences [65] used parts of speech (POS) tagging on corpus of ambiguous words including “always,” “every,” “none,” “certainly,” “therefore,” “good,” “often,” “rejected,” “such as, “they,” and “those.” But the tool does not provide detailed description of those words or sentences that were ambiguous or created ambiguity. Similarly, a framework for NL transition to controlled NL (CNL) was designed in a way to lessen the complexity of ambiguity formed in a sentence [66]. The aim of this work was to avoid inducting ambiguity in SRS document at first place. The prototype performed lexical, semantic, and syntactic analysis concerning SBVR (semantic business vocabulary and rules). A framework was designed using POS tagging for detection of syntactic and semantic ambiguity in SRS [15]. POS tags words of sentences to equivalence tagger, and then ambiguity detector, based on seven rules of ambiguity classification, classify ambiguity. As the framework was at its early stages, it required implementation in a functioning system. It was also observed that human requires a lot of knowledge to detect ambiguity in a sentence.

For evaluation of this approach, nocuous ambiguity identification (NAI) prototype tool was used, but to cover full aspects of ambiguity, more heuristics are required [62]. POS tags words of sentences to equivalence tagger, and then ambiguity detector, based on seven rules of ambiguity classification, classify ambiguity. A framework was designed to categorize ambiguity occur in interviews during requirements elicitation [67]. The framework operates on four factors including unclear requirements, misunderstood requirements, correct and incorrect disambiguation of requirements. The work also shows how ambiguity is linked to the knowledge known to the customer but does not pass to the analyst during interviews.

Similarly, POS tagging is used to detect syntax and syntactic ambiguities of SRS written in NL [68]. An experiment conducted to cross-check the detection of ambiguity, with the help of an automated ambiguity detector tool. The tool has its own limitations like limited file format, that is, text file, focused on two types of ambiguity, and did not record or save any activity. It is also observed that human requires a lot of knowledge to detect ambiguity in a sentence.

The written requirements in SRS document were automatically translated to SBVR using SR-Elicitor [62]. The tool based on SBVR was developed to help software engineers in recording and transforming requirements written in NL to SBVR SRS. Although, SR-Elicitor was not meant to be used for object-oriented concepts like classes and instances, but it was designed for enhancing communication business rules among business community. In NLP, the modern approach of object-oriented approach “OpenNLP” was used that gained much popularity [69]. In this approach, POS tagging was used on NL statements to produce SRS document. Similarly, set of cues were identified in the linguistic expressions of the customers that led towards ambiguity [17]. Interviews of customer and analyst were performed, and ambiguous speech fragments were isolated. These cues were used as a reference guide to detect ambiguity, by the analyst.

Literature has shown that different methods such as unified modelling language (UML), ontology-based, and NLP have been used for resolving ambiguity problems. There is less work done on automatically detecting ambiguity in SRS written in NL, using POS technique. Software Requirement Ambiguity Avoidance Framework (SRAAF) [70] was designed to support requirements engineer for writing unambiguous requirements by selecting well-suited elicitation technique. The framework, conducted with W6H technique, was based on evaluation of different attributes. Project features, attributes of stakeholders and requirements engineer, and W6H technique helped in the selection of elicitation technique. It was focused to avoid ambiguities even before writing requirements in the SRS document.  Table 3 shows year-wise contribution of previous work along with the targeted area of requirements elicitation and limitations.

Table 3 summarizes literature on requirements ambiguity by highlighting the contribution of the work, targeted area of ambiguity, ambiguity handling level, and limitation of the work.

#### 2.1.2. Gamification in Requirements' Elicitation

Visual techniques are used for requirements elicitation to support the process in an interactive way. ELICA the ELICitation Aid [72] tool records the intentions of speaker with the help of interactive visualization and used analytical tone and emotions to gather requirements from the database of existing documents. The major limitation of ELICA is absence of user participation throughout the process. AirT [73] uses storyboards to elicit the feedback of user and send frequent reminders for using the tool. Some of its limitations are infeasibility with the resources of the project and timeline due to which some of the requirements get postponed to later versions. It is observed that more than one elicitation techniques have been used to get the requirements. Researchers have developed more interactive interfaces for increasing user engagement during elicitation, so they may get required information from the user. One of the most recent interactive ways to get user engage in the system is “gamification” [32, 71], which is used during requirements elicitation.

Gamification is used in the elicitation process [74], in which few aspects are gamified, yet there are many to be explored. iThink [34] developed in 2012 is a gamified tool used to enhance the participation and collaboration of stakeholders. It is based on the concept of creative thinking behind the idea of gamification, that is, *six thinking hats*. Upon generation of a new requirement and refinement of any requirements, players are rewarded. The users have different roles including player and project manager. A project manager creates a project but does not consider as a player, thus does not get any rewards. iThink is implemented in outsystems agile platform. The evaluation of iThink is done based on two case studies, and it was concluded that although it helps to engage and motivate the users, but it has few drawbacks such as dependency of how ideas are generated, generalization of results due to limited test sample.

Similarly, Requirement Elicitation and Verification Integrated in Social Environment (REVISE) [36], idea is proposed to maximize the knowledge sharing and collaboration among project team members. The idea behind REVISE is based on CARE principles of create, ask for review, review, and extend. Three roles were involved in the system including creator, reviewer, and customer. All stakeholders can add new requirements and able to trace them. Scores were used to reward the players, but it was concluded that other gaming elements such as leaderboard, badges, and profile could be used. REVISE does not use any requirements document as only theoretical framework of REVISE is given without any further implementation.

The lack of user involvement in the system yields poor requirements and system performance. In this context, a gamified requirement engineering model GREM [33] is designed to use gamification in requirements elicitation. The purpose is to involve customers in the elicitation process so that the performance of system could be improved. GREM is based on three variables, that is, gamification, stakeholder's engagement, and performance. Dichotomous variable, Reiss Profile, and Positive and Negative Affect Schedule (PANAS) are used to measure variables, motivation, and emotions respectively. PBL, levels, activity feeds, and challenges are used in the gaming platform, whereas evaluation was done under a controlled experiment conducted on 12 employees of a company. The employees are categorized based on motivation, expertise, and gender. Although, more experiments to represent requirements are required by focusing stakeholder's engagement to the system, yet gamification helped in improving the quality, creativity, and productivity of the system. Collaboration and communication among stakeholders are reduced, as reported by the participants. However, the choice of gaming elements has an impact on system performance as well as stakeholder's engagement.

In a similar system [58], focused on stakeholder's engagement in requirements elicitation, a scenario-based RE gamification platform is developed having two variables, that is, motivation and expertise of stakeholder. Three dimensions are defined to engage user to the system, including emotions, cognition, and behaviour. Almost seventeen gaming elements are used to measure these variables; Reiss profile, PANAS, and Flow Shor Scale (FSS) are used to measure the emotions. For evaluation of the platform, experiments are conducted on an IT firm, and it was observed that the behaviour created more statistical difference than the emotions. The stakeholders who enjoy using gaming elements, found to be more active in requirements production, hence user engagement is quite high during the process. Furthermore, gamification helps to boost user performance, which derived in changing behavioural dimension. The limitation of this platform is difficulty in keeping track of user stories because of having too many people involved in the system, small size of the sample, limited number of interested employees who took part in the experiment. In other work, for stakeholder's engagement in RE and prioritization of requirements, DMGame [75] is used. DMGame uses analytic hierarchy process (AHP) and genetic algorithms for requirements prioritization. There are three main roles involved in the system including supervisor, opinion provider, and negotiator. The tool use gaming elements such as progress, time pressure, and pontification to support collaborative requirements prioritization. The tool is validated on three industrial case studies taken from the SUPERSEDE project.

A generic framework Agon is designed to model, analyse, and fulfil acceptance requirements using gamification [76]. Agon uses four models namely acceptance model (AM), tactical model (TM), gamification model (GM), and user context model (UCM) at three different levels. AM, TM, and GM are designed by extending nonfunctional requirements framework (NFR), and by using context dimension trees UCM is designed. Agon is validated on a meeting scheduler example with 270 goals and 376 relations among operations, refinements, and contributions. It used popular game elements points, leaderboard, and ranking. The evaluation of the framework is not thorough as it was performed on already developed example. Owing to its complex nature, it is concluded that more real case studies were required to validate the generality, versatility, and utility of the framework. Agon was later compared with motivational antecedents framework (MAF) on same case study of meeting schedular [77]. The foundation of MAF is laid on human and organizational behaviour, whereas Agon is designed on the principles of software engineering which advocates aspects of user, software, cognition, and psychology for user engagement.

In other work, a meta-model for Agon [78] is described supported by the gamification, using a Systematic Acceptance Requirements Analysis Framework (SARAF). The framework supports analysis and design of software systems. Participatory Architectural Change Management in ATM Systems (PACAS) is introduced for the air traffic management (ATM) system. It is also based on psychological strategies and gaming solutions for serious problems. According to the preliminary evidence collected from the nonexperts and experts, that is, students and experts of gamification and RE, Agon was a useful framework.

For designing gamified solutions, factors like motivation and acceptance are needed and for this purpose, stakeholder's participation is required throughout the process. In a similar work [79], set of key requirements for designing a gamified solution is discussed. The two major parts of the system are Agon framework and design thinking. The analysis of different models and case studies including DMGame and SUPERSEDE [75] are performed to identify key requirements.  Table 4 covers year-wise work presented in literature on gamification in requirements elicitation, gaming elements used by the studies, and limitations of the work.

Gamification solutions in requirements elicitation depends hugely on the selection and use of game elements. Previous studies show that game elements are used for engaging users to the system. Other than the game elements presented in Table 4, Table 5 presents mapping of more game elements used in gamified systems used for requirements elicitation.

In Table 5, 20 gaming elements are identified from the relevant studies on requirements elicitation.  Figure 3 shows the use of each game element in selected studies.

In Figure 3, the game elements from Table 5 are shown with frequency of use in different related studies. According to the literature, points are frequently used in requirements elicitation.

## 3. Discussion

A gamification based RE requires a lot of analysis, awareness of participation, difficulty of finding active users and others. Several studies have also revealed the negative impact of selecting less sample size on overall project. The issues in practice such as lack of technology support, unreliable results of such platforms, and problems of evaluation are still there. Multiple studies have reported the limitations of using gamification platforms in elicitation, such as less visual appeal [34], ineffective results, absence of conceptual foundations [36], invalidity of developed solution [1], and biasness of results [82].  Figure 3 presents most used game elements in requirements elicitation which are points, leaderboards, and badges with 45%, 35%, and 25% frequency of use respectively. On the contrary, awards, rewards, levels, game roles, and medals occurred 20%, 15%, 10% and 5%, respectively. It is observed that some game elements like challenges, rules, paths, goal, feedback, avatars, scores, and activity feed have a limited use as compared to PBL.

## 4. Conclusion and Future Work

Requirements ambiguity is a critical challenge in NL that occurs majorly due to lack of understanding, undefined scope, and unclear context of the system. In elicitation, gamification is highly effective for engagement and interaction between the stakeholders. Previously, there are no studies available that reduce ambiguity in NL-based requirements with the help of gamification. In this review, requirement ambiguity is discussed with the classification of ambiguity types. We have discussed five classes of ambiguity including lexical, semantic, syntactic, pragmatic, and language errors, nine relevant requirements ambiguity studies, three visual requirements elicitation techniques, 20 game elements, and eight gamification elicitation techniques. It is observed that the most used game elements during elicitation are PBL, but the use of game elements is a design decision that largely depends on roles involved in the system. Furthermore, based on the findings of this review, a framework will be proposed to help the project team and users to elicit requirements and reduce the ambiguity at the time of elicitation. We are currently working on the development of the gamified tool followed by its industry evaluation. In future, the enhancement of tool can be done by involving more user roles to the system, exploring more design options with other classes of ambiguity, in different types of projects.

## Figures and Tables

**Figure 1:** Types of natural language ambiguities.

**Figure 2:** Methodology of the review.

**Figure 3:** Frequency of using game elements.

**Table 1:** Difference between a digital game and gamification.

Digital game	Gamification
Rules and objectives derive games	Reward and points are deriving forces
Result is winning or losing	Losing is not possible
Complex and costly	Not complex and costly
Based on some story, content-based	Addition of gaming features without content

**Table 2:** Game elements used in gamification.

Game elements	Description
Awards/rewards	Given on completion of a task or behaviour
Points	Points are given when a certain task is completed
Badges	Badges represents of achievements
Leaderboard	Leaderboard presents ranking of different players
Ranks	Ranks represents increase in a competence level of the players
Levels	Levels are achieved after gaining certain number of points
Quests	Quest represents a story-based task that must be completed by the player
Bets	Bets are like estimation where player bets on certain event
Avatars	Avatar represents a virtual character of a player having personalized attributes and interests
Stories	Stories represent dramatic sequence or narrative to stimulate emotions of the players

**Table 3:** Related work on ambiguity in requirements elicitation.

Ref.	Year	Contribution	Targeted ambiguity type	Ambiguity handling level	Limitations
[5]	2008	The proposed work checks lexical ambiguity using algorithm in requirements document and validate the solution using algorithm	Identifying lexical ambiguity in NL-based written requirements	Ambiguity detection	Insufficiency of solution for lexical ambiguity in a sentence
[65]	2010	The system uses machine learning algorithm for ambiguity detection in requirements document. The algorithm, along with NAI tool, uses heuristic evaluation to identify the type of ambiguity	Identifying nocuous ambiguity in NL-based requirements document	Ambiguity detection	Selected heuristic evaluation was insufficient to explore different aspects of ambiguity, tool validity was unclear, and the tool supported only coordination ambiguity
[71]	2011	A tool SR-elicitor was used with SBVR to translate the SRS to SBVR. It generates software models with the help of mathematical expressions	Transformation of NL-based requirements of SRS to SBVR	Ambiguity detection and reduction	The tool does not support concept of OO such as instances, classes.
[69]	2012	A tool to detect ambiguity in words was developed using POS tagger	Detection of lexical, syntactic, and semantic ambiguity of the SRS document	Ambiguity detection	The tool does not provide detailed description of the ambiguous words
[17]	2016	The work was based on identification of cues in customer's expressions, from speech of fragments of the conversation between customer and analyst during interviews. These cues were used for ambiguity detection	Detection of ambiguity in elicited requirements during the interviews	Ambiguity detection	The proposed approach does not work well if analyst is not known to ambiguity
[68]		The proposed work was based on categorization of ambiguity in interviews. A theoretical framework was designed for this purpose. To study this phenomenon, a set of 34 analyst-customer interviews were conducted and analyzed	Categorization of ambiguity in elicited requirements gathered during interviews	Ambiguity detection and categorization	
[15]	2017	A framework for ambiguity detection was developed using POS tagging along with ambiguity detector tool to tag the ambiguous words in a sentence	Detection of syntactic and semantic ambiguity of NL-based requirements of SRS document	Ambiguity detection	The tool was in its early stages, hence implementation of framework in a functioning system was required
[68]	2018	A tool using POS tagging for detection of ambiguity in requirements, was developed	Detection of syntax and syntactic ambiguity in NL-based requirements of SRS document	Ambiguity detection	The tool was limited to accept the file only in.txt format, does not save any record, much knowledge of ambiguity was required
[70]	2019	A tool SRAAF based on W6H technique was developed to write ambiguity-free requirements, with the help of selecting appropriate elicitation technique(s)	Avoidance of ambiguity before writing statements in SRS document, and selection of suitable elicitation technique	Ambiguity reduction	The tool does not support advanced NLP technology of W6H techniques, it is not fully implemented and currently not available
[66]	2020	A prototype for NL based on CNL transitioning was developed for analysis of ambiguity in SRS document	Avoidance of lexical, semantic, and syntactic ambiguity in NL-based requirements of SRS document	Ambiguity reduction	The tool used only one expert to create the sample data which does not represent set of population of experts, another limitation is less experienced of the expert

**Table 4:** Related work on gamification in requirements elicitation.

Ref.	Year	RE gamification	Focus of the work	Gaming elements	Limitations
[34]	2012 iThink	A game-based tool for collaboration and to gather requirements. It used a creative thinking technique “six thinking hats”	Collaboration	Rewards	Limited test sample, problem in generalization of data
[36]	2015REVISE	A tool developed for requirements elicitation from stakeholders and verification	Requirements gathering, requirements verification	Score, badges, and leaderboards	Not tested and evaluated
[80]	2015REfine	For cloud centric RE in software product organization, a prototype tool was used to engage the stakeholders in RE	Stakeholder's engagement	Leaderboards, points, and roles	Less attractive system features, inexperienced team, issues in merging user needs to the system
[33]	2016GREM	A model helps to engage stakeholders to RE and helps in improving the performance of RE with gamification	Stakeholder's engagement	PBL, levels, challenges, and activity feeds	Reduced stakeholder's collaboration and communication having negative impact on the system, not evaluated for stakeholder's engagement
[35]	2017no name	With the help of REfine tool in crowd centeric RE engages stakeholders to the process of RE	Stakeholder's engagement	Roles, points, leaderboards, group formation, and exploration	Not a “one size fits all' solution, negatively influence the reliability of requirements, limited sample size for validation
[75]	2017DMGame	A tool to involve and motivate stakeholders in prioritization of requirements for decision making	Stakeholder's engagement, requirements prioritization	Progress, time pressure, and pointsification	-
[81]	2018No name	A gamified requirement inspection ring-i process was proposed to allow users and other stakeholders for verification of i∗models	Requirements inspection, verification	Rules, goal, and feedback system	Inconsistent model, unclear idea, no empirical evaluation
[82]	2019GARUSO	An approach to involve stakeholders from outside of organization in RE process	Stakeholder's involvement	Points and levels	Doubtful quality of resulting requirements, biased results, and other certain limitations

**Table 5:** Game elements for requirements elicitation.

Game elements	2012 [34]	2015 [36]	2015 [80]	2016 [33]	2016 [58]	2016 [76]	2017 [77]	2017 [78]	2017 [35]	2017 [75]	2018 [81]	2019 [82]
Awards/rewards	Yes					Yes	Yes	Yes				
Points			Yes	Yes	Yes	Yes	Yes	Yes	Yes	Yes		Yes
Scores		Yes										
Badges		Yes		Yes		Yes		Yes	Yes			
Leaderboard		Yes	Yes	Yes	Yes	Yes		Yes	Yes			
Rank												
Levels				Yes		Yes		Yes				Yes
Game roles			Yes		Yes	Yes		Yes				
Medal			Yes		Yes	Yes	Yes					
Quest												
Bet												
Avatars								Yes				
Story												
Challenges				Yes				Yes				
Activity feed				Yes								
Goal				Yes			Yes				Yes	
Rules				Yes							Yes	
Feedback				Yes						Yes	Yes	
Paths							Yes	Yes				

## Data Availability

The graph, figures, and tables' data used to support the findings of this study are included within the article.
